The article "Availability Bias and the COVID-19 Pandemic: A Case Study of Legionella Pneumonia" was published in 2022. Journal: Cureus.

# Availability Bias and the COVID-19 Pandemic: A Case Study of Legionella Pneumonia

**DOI:** 10.7759/cureus.25846

**Published:** 2022-06-11

**Authors:** Kwaku Kyere, Taiwo O Aremu, Oluwafemi A Ajibola

**Affiliations:** 1 Department of Medicine, Nuvance Health, Vassar Brothers Medical Center, Poughkeepsie, USA; 2 Department of Pharmaceutical Care & Health Systems, College of Pharmacy, University of Minnesota, Minneapolis, USA; 3 Division of Environmental Health Sciences, School of Public Health, University of Minnesota, Minneapolis, USA

**Keywords:** sars-cov-2, coronavirus disease 2019 (covid-19), availability heuristic, legionellosis, availability bias, covid-19 pandemic, legionella pneumonia, cognitive biases

## Abstract

Cognitive biases, such as the availability heuristic or availability bias, can inadvertently affect patient outcomes. These biases may be magnified during times of heightened awareness of a particular disease. Failure to identify cognitive biases when managing patients during the coronavirus disease 2019 (COVID-19) pandemic can delay the institution of the right treatment option and result in poor health outcomes. We present a case of delayed diagnosis of Legionella pneumonia due to COVID-19-related availability bias. We discuss some methods to mitigate the effects of this bias and the importance of challenging trainees to recognize these pitfalls in medical training.

## Introduction

A new and severe respiratory infection of unknown etiology, named coronavirus disease 2019 (COVID-19), was first reported in Wuhan, Hubei Province of China, in December 2019. This was the beginning of a pandemic affecting virtually every country on the planet at an alarming rate with a significant death toll. The clinical presentation of COVID-19 is marked by flu-like symptoms, including fever, cough, malaise, and fatigue. Other less frequently reported symptoms to include loss of sense and taste and smell, nausea, and diarrhea. Chest X-ray and Computerized Tomography (CT) often show patchy bilateral infiltrates, a radiological characteristic typically associated with atypical pneumonia. A subset of patients develops acute respiratory distress syndrome (ARDS), requiring intubation and mechanical ventilation, with or without septic shock, and multiorgan system failure. The causative organism is a coronavirus formally named SARS-CoV-2, which has significant homology to SARS CoV-1, responsible for the severe acute respiratory syndrome (SARS) of 2002. Both pathogens are believed to be zoonotic organisms originating from animal reservoirs and gained human-to-human transmissibility [1].

*Legionella pneumophila *was identified in 1979 as the causative pathogen of previously unidentified pneumonia after an outbreak among attendees at a convention of the American Legion three years earlier [2-4]. Since then, it has been estimated that about 8,000-18,000 Americans have been hospitalized with legionellosis annually [5]. The disease occurs following the inhalation of aerosolized droplets containing the bacteria or after aspiration of contaminated water [6]. Two distinct disease entities can result from legionellosis: Legionnaires' disease, a severe form of pneumonia resulting in multiorgan system involvement/failure, and Pontiac fever, a more benign, self-limited, flu-like illness [3,7]. Legionellosis is among the group of pneumonia classified as atypical pneumonia, similar to the pattern of pulmonary disease seen in COVID-19. Symptoms include fever, nonproductive cough, headache, myalgias, rigors, shortness of breath, and diarrhea [8]. Hyponatremia has been associated with legionellosis [9]. A urine antigen test is accessible for rapid diagnosis.

As one can imagine, an inaccurate initial diagnosis can result in mismanagement and cause unintended harm to patients. The role of cognitive biases, such as anchoring, overconfidence bias, premature closure, confirmation bias, and availability bias, as sources of flawed medical decision-making and medical errors are well established in the literature [10,11]. Clinicians' awareness of these faulty mental frameworks can minimize their adverse effects. This need is heightened when ideal conditions exist for these heuristics to fail us, such as during a pandemic when quick decision-making is often required.

## Case presentation

A 56-year-old man presented to the emergency department with four days history of fevers and shortness of breath during the height of the COVID-19 pandemic. He disclosed exposure to known cases of COVID-19. There was no history of cough, chest pain, nausea, or vomiting; however, the patient had extreme fatigue. He has a past medical history of diabetes mellitus, hyperlipidemia, and hypertension. There was no history of smoking. The vital signs on presentation showed a maximum temperature of 104.0 degrees Fahrenheit, a heart rate of 128 beats per minute, a respiratory rate of 28 breaths per minute, and an oxygen saturation of 92% on room air. The physical examination was remarkable for diminished breath sounds in the left lower lobe. 

The initial laboratory studies showed leukocytosis with lymphopenia, normal hemoglobin level, and thrombocytopenia. There were elevated D-dimer, ferritin, C-reactive protein (CRP), procalcitonin, and lactic acid levels. The creatinine level was normal, but the patient had significant hyponatremia (Table 1).

**Table 1:** Laboratory values

Laboratory Parameter	Patient’s value	Reference range
White Blood Cell (WBC) count	11.9 k/µL	4.5–11.0 k/µL
Hemoglobin	13 g/dL	12–16 g/dL
Platelet count	130 k/mm^3^	150–400 k/mm^3^
D-dimer	2112 ng/mL D-DU	0–230 ng/mL D-DU
Ferritin	4820 ng/mL	24–370 ng/mL
C-reactive protein (CRP)	28.5 mg/L	0–8 mg/L
Procalcitonin	8.6 ng/mL	≤ 0.08 ng/mL
Lactic acid	2.7 mmol/L	≤2.0 mmol/L
Sodium	127 mmol/L	136–145 mmol/L

The rapid COVID-19 test on admission was negative.

The electrocardiogram (EKG) showed sinus tachycardia (Figure 1).

**Figure 1:** Electrocardiogram (EKG) showing signs of sinus tachycardia

Chest X-ray showed an ill-defined pulmonary infiltrate in the lower lobe of the left lung that suggested pneumonia (Figure 2).

**Figure 2:** Chest X-ray showing pulmonary infiltrates on the left The blue arrow indicates an area of ill-defined infiltrates in the lower lobe of the left lung.

A CT angiogram of the chest was obtained following an elevated d-dimer, a high pre-test probability of pulmonary embolism (PE). This was negative for PE but showed an extensive left lower lobe airspace consolidation suspicious for lobar pneumonia (Figure 3).

**Figure 3:** CT angiogram of the chest The red arrow indicates an area of airspace consolidation on the lower lobe of the left lung

The patient was initially started on ceftriaxone and azithromycin for possible bacteria pneumonia. However, the following day, his condition deteriorated with persistent fevers and hypoxemia, necessitating broadening antibiotics to vancomycin, piperacillin-tazobactam, and azithromycin. Repeat rapid COVID-19 test and a COVID-19 PCR test were conducted, both of which were negative. The patient was maintained in continued isolation with droplet and contact precautions and required personal protective equipment to enable routine evaluation. On day two of admission, due to persistent hyponatremia, a urine antigen test for Legionella was requested and returned positive. Given the three negative COVID-19 test results and confirmed legionella pneumonia, isolation was discontinued, and antibiotics were de-escalated to azithromycin. Although he required significant oxygen support before COVID-19 was ruled out, non-invasive positive pressure ventilation and high flow nasal cannula were not attempted based on clinical guidelines.

Over time, his oxygen requirements decreased with appropriate antibiotic therapy. He had slow but steady improvement, and by day seven of hospitalization, he was weaned off oxygen and discharged home.

## Discussion

The COVID-19 pandemic has had and will likely continue to have a profound psychological impact on the United States and the rest of the world. Many generations will become aware of this global event and its devastating effects from their family, simulated movies, literature, etc. Another unforeseen adversary for physicians at the forefront of this battle against SARS-CoV-2 is cognitive bias/error, including anchoring, overconfidence bias, premature closure, confirmation bias, and availability bias [10,11].

Mamede et al. reported the effects of availability bias among resident physicians in 2010 [11]. When primed to think of a particular diagnosis, physicians were more likely to make the primed diagnosis given a similar presentation of an otherwise unrelated illness. During the early phase of the COVID-19 pandemic, many patients admitted to our hospital had respiratory disease with symptoms such as fever, cough, lethargy, etc. It is important to note that not all these patients had COVID-19. At any other time, clinicians might have been more likely to consider other diagnoses. However, due to the nature of COVID-19, particularly the risk it poses to patients and caregivers if not correctly diagnosed, there is often a very high index of suspicion for this diagnosis collectively. COVID-19 can become a highly available diagnosis, get anchored, and potentially lead to poor outcomes. Moreover, it can lead to inappropriate use of scarce personal protective equipment (PPE).

Our patient exhibited many of the symptoms and diagnostic findings associated with COVID-19. Furthermore, he had come in contact with known cases of COVID-19 and was deemed to have a high pretest probability of having contracted the disease. Although he tested negative three times for COVID-19, due to the powerful effects of anchoring, the diagnosis of COVID-19 remained high on the differential as it arguably should be. It is equally important to recognize that other diagnoses are possible. This need for a heightened awareness of alternative diagnoses is essential during times when there is a high propensity to fall into the traps of availability bias. Domination of the socio-medical consciousness made COVID-19 a very available diagnosis, which can be problematic even among highly experienced clinicians.

It is known that clinicians are more prone to biases when using non-analytical reasoning, i.e., the type of reasoning that develops with pattern recognition and, coincidentally, with clinician experience [11]. The literature has reported that methods that utilize a more analytic approach may reduce the effects of availability bias and potentially other biases as well. In our case, analyzing the patient's particular presentation took into account his hyponatremia, which has been associated with Legionella pneumonia [9] and ultimately led to the correct diagnosis. Furthermore, metacognition, that is, thinking about one's own thoughts/cognitive processes, has also been shown to mitigate some of the effects of cognitive biases in medicine.

Lastly, the time-tested art of generating a differential diagnosis is immensely helpful in preventing many cognitive lapses that may lead to inaccurate decision-making in the care of all patients [12]. Generating differential diagnoses is a simple and effective tool taught in all medical schools and residency programs in the United States. We also believe that it is indispensable both during *business as usual* and in times of amplified biases. Its very nature forces us to consider other alternatives even when we feel we have a diagnosis. It encourages us to check our thoughts and decisions, which is indispensable when working in the busy, fast-paced world of medicine. It compels us to slow down and reason.

## Conclusions

As we continue to battle the COVID-19 pandemic, physicians should be aware of availability bias and potential biases that may inadvertently affect patient outcomes. Cognitive biases such as the availability bias are significant contributors to poor patient outcomes, including morbidity and mortality; hence they constitute a concept of clinical importance. Utilizing metacognition and generating a differential diagnosis with a more analytic approach can help clinicians minimize these biases, take better care of their patients and improve overall health outcomes.
